The article "RGB and HSV quantitative analysis of autofluorescence bronchoscopy used for characterization and identification of bronchopulmonary cancer" was retracted in 2020. Reason: duplicate publication.

# RGB and HSV quantitative analysis of autofluorescence bronchoscopy used for characterization and identification of bronchopulmonary cancer

**DOI:** 10.1002/cam4.831

**Published:** 2016-10-05

**Authors:** Xiaoxuan Zheng, Hongkai Xiong, Yong Li, Baohui Han, Jiayuan Sun

**Affiliations:** ^1^ Department of EndoscopyShanghai Chest Hospital, Shanghai Jiao Tong UniversityShanghai 200030China; ^2^ Department of Electronic EngineeringShanghai Jiao Tong UniversityShanghai 200240China; ^3^ Department of pulmonary medicineShanghai Chest Hospital, Shanghai Jiao Tong UniversityShanghai 200030China

**Keywords:** Autofluorescence bronchoscopy, bronchopulmonary cancer, diagnosis, medical image processing, white light bronchoscopy

## Abstract

Autofluorescence bronchoscopy (AFB) shows good sensitivity in detecting dysplasia and bronchopulmonary cancer. However, the poor specificity of AFB would lead to excessive biopsy. The aim of the study is to establish a more effective quantitative method (optimal identification index and reference value) for characterizing the AFB images within the region of interest and discuss AFB's significance in the diagnosis of central‐type lung cancer. A total of 218 suspected lung cancer patients were enrolled in this study. A quantitative analysis based on color space (red, green, blue[RGB] and HSV system) was conducted and the result was compared with the final diagnosis obtained by the pathology of biopsy. Cases were divided into different groups according to the pathological diagnosis of normal bronchial mucosa, inflammation, low‐grade preinvasive (LGD), high‐grade preinvasive (HGD), and invasive cancer. Quantitative analyses in multi‐color spaces for the lesions showed by AFB images were conducted by software MATLAB. Finally, there is statistical significance among the different groups in some parameter in RGB and HSV system. So, both RGB and HSV quantitative analysis of autofluorescence bronchoscopy are useful to define benign and malignant diseases, which can objectively guide the bronchoscopist in selecting sites for biopsy with good pathologic correlation.

## Introduction

Bronchopulmonary cancer is one of the most common malignancies in the world, and currently, it is also the main cause leading to death with tumor in the world. Both central‐type early lung cancer (CELC) and peripheral cancer have a high incidence. The prognosis of lung cancer is closely related to tumor stage 1, 2, 3. Therefore, early detection, early diagnosis, and early treatment of lung cancer are the key to improving the prognosis of patients with lung cancer.

Bronchoscopy and sputum cytology are main clinical methods to detect CELC, while the positive rate of sputum cytology is very low, and bronchoscopy can only increase the discovery rate of CELC slightly compared with sputum cytology 4. In general, CELC cases show only minor changes in the bronchial mucosa using white light bronchoscope (WLB). It is even more difficult to detect moderate‐to‐severe dysplasia using WLB by even an experienced bronchoscopist 5.Therefore, there is an urgent need to find new means for early detection, locating and diagnosing lung cancer, thereby improving prognosis of patients and reducing lung cancer mortality.

Autofluorescence bronchoscopy (AFB) can significantly improve early diagnosis sensitivity of lung cancer and precancerous lesions 6. However, the specificity of AFB may be its limitations; because red fluorescence also shows in cases of bronchial mucosal inflammation, inflammatory granuloma, scar tissue, and mucosal injury, which can easily be confused with precancerous lesions, carcinoma in situ (CIS), and invasive carcinoma 7.The current qualitative diagnostic method of determining the results only by color changes has greater limitation, which is not conducive for precise judgment in practical operation.

Therefore, we hope to obtain more intuitive numerical information by analysis and quanititation of color information to more accurately guide our clinical procedures, and to quantify the fluorescence intensity of different pathological stages in the course of lung cancer so that this method exerts larger values in early diagnosis and assessment of the degree of local canceration.

## Patients and Methods

### Patients

This was a retrospective study of patients who underwent WLB associated with AFB at Shanghai Chest Hospital from April 2012 to January 2014. The work was approved by ethical committees of Shanghai Chest Hospital. All patients were informed and signed the informed consent before the examination.WLB and AFB were performed according to the following guidelines: (1) Patients who had recently developed central‐type lung cancer or were suspected to be affected by lung cancer due to changes in existing symptoms, such as cough, expectoration, hemoptysis, hoarseness, body weight loss, etc.; (2) clinical suspicion of central‐type lung cancer due to abnormal sputum cytology as well as lung‐occupying lesion; (3) pulmonary atelectasis or flake shadows suggested by imaging examination; (4) Informed written consent was obtained from all patients and the institutional review board approved this study (KS10‐03); and (5) no contraindication to the procedure. There were exclusion criteria for the study: (1) Patients who had history of bronchoscopy and underwent biopsy and brushing biopsy recently; (2) those who had bronchoscopy contraindications (active and massive hemoptysis, unstable angina pectoris, allergic to anesthetics, etc.); (3) those who had undergone cytotoxic chemotherapy within 6 months; (4) those who had taken photosensitizing drugs within 3 months.

### WLB and AFB examination

This study adopted BF‐F260 electronic AFB (Japan, Olympus Corporation) that has both WLB and AFB function and can be switched between white light mode and autofluorescence mode. Firstly, glottis, airway carina, left and right main bronchi, and lobar, segmental and subsegmental bronchi were examined under white light; tracheal rings, mucosa, blood vessels, secretions, neoformation, etc. were observed and followed by AFB. Finally, biopsy was always done if necessary according to operator's judgment.

### WLB and AFB image characteristics for lesions

Under ordinary white light, the visible lesions were divided into three levels 8: WLB I: congenital anatomic abnormality, compressive lesion, simple broadened bronchial bridge, normal color of mucosa, without hyperemia and edema; WLBII: mucosal hyperemia, edema, thickened, change in color, vessel convergence or distortion; WLBIII: granular‐like changes in mucosa or presence of apparent neoformation. WLBII and WLBIII were defined as the abnormal findings under WLB. Under the autofluorescent state, the visible lesions were also divided into three levels: AFBI: green mucosa; AFBII: the color of mucosa slightly changed to pale pink or brown; AFBIII: the color of mucosa changed to typical red or red purple. AFBII and AFBIII were defined as the abnormal findings under AFB. Both WLB and AFB were conducted by two experienced physicians who were blinded to the pathological results and graded the images. If the grading was not consistent, it was concluded through discussion with the chief physician.

### Evaluation of pathological results

Pathological diagnosis was made by two experienced pathologists who were blinded to the grading by operating physicians. If the diagnosis was not consistent, it was concluded through discussion with the chief physician. The diagnosis following discussion was the final conclusion.

The pathological diagnoses were divided into invasive carcinoma, CIS, severe dysplasia, moderate dysplasia, mild dysplasia, hyperplasia, squamous metaplasia, inflammation, and normal cell 9. The pathological diagnosis of severe dysplasia and CIS were defined as high‐grade preinvasive (HGD); hyperplasia, squamous metaplasia, mild and moderate dysplasia were defined as low‐grade preinvasive(LGD). Pathological diagnosis of HGD and invasive carcinoma were defined as positive diagnosis; normal mucosa, inflammation, and LGD were defined as negative diagnosis 9.

### Quantitative analysis of AFB images

AFB images were collected and stored by the same set of system, and processed by MATLAB software (R2012b version, MathWorks Inc., Natick, USA) in the same computer. 16 × 16 pixel target regions in the center and two edges of the lesion were measured, and the average values of the three regions was taken as the final data, which was analyzed by the software to obtain R, G, B, R/G, R/B, G/B, H ,S, and V values. The conversion formula of HSV (hue, saturation, value) and RGB (red, green, blue) values is shown in Formula 1^10^:

$$\begin{array}{cc} & \left\{\begin{array}{c} V=T_{\max}\\ S=\left\{\begin{array}{cc} 0, & \text{if}T_{\max}=0\\ \frac{T_{\max}-T_{\min}}{T_{\max}}=1-\frac{T_{\min}}{T_{\max}}, & \text{otherwise} \end{array}\right.\\ H^{\prime }=\left\{\begin{array}{c} 60\times \frac{G-B}{T_{\max}-T_{\min}},\\ \text{if}\left(s\neq 0\right)\;\text{and}\;\left(T_{\max}=R\right)\\ 60\times \left(\frac{B-R}{T_{\max}-T_{\min}}+2\right),\\ \text{if}\left(S\neq 0\right)\;\text{and}\;\left(T_{\max}=G\right)\\ 60\times \left(\frac{R-G}{T_{\max}-T_{\min}}+4\right)\\ \text{if}\left(S\neq 0\right)\;\text{and}\;\left(T_{\max}=B\right) \end{array}\right.\\ H=\left\{\begin{array}{cc} H^{\prime }, & \text{if}H^{\prime }\geq 0\\ H^{\prime }+360, & otherwise \end{array}\right. \end{array}\right. \end{array}$$

Formula 1 Equation RGB and HSV values conversion formula.

### Statistical analysis

SPSS 11.5 (SPSSInc., Chicago, IL, USA) software was used to process data; measurement data was expressed as mean ± standard deviation (Mean ± SD), and numeration data was expressed as percentage. LSD method of one‐way analysis of variance (ANOVA) was used to compare data between the groups. The chi‐square test or Fischer's exact test was performed, when appropriate, for categorical variables.

## Results

### Pathology results

A total of 218 cases with 1208 effective pathological specimens (5.5 on average) were obtained. All biopsy specimens used in this study had definite pathological diagnosis.

The final diagnosis is shown in Table 1. The representative cases of each groups are shown in Figure 1.

**Table 1:** Pathological diagnosis of bronchoscopy biopsy

Pathological diagnosis	Number of cases(*n*)	Percentage(%)
Squamous cell carcinoma	72	33.0
Adenocarcinoma	31	14.2
Small cell carcinoma	31	14.2
Undifferentiated carcinoma	16	7.3
HGD	14	6.4
LGD	9	4.1
Normal	13	6.0
Inflammation	32	14.7
Total	218	100

HGD, high‐grade preinvasive; LGD, low‐grade preinvasive.

**Figure 1:** Representative cases of each group (A1, B1, C1): Representative white light bronchoscope (WLB), autofluorescence bronchoscopy (AFB) imaging and red, green, blue (RGB) histogram analysis of normal bronchial mucosa. (A2, B2, C2): Representative WLB,AFB imaging and RGB histogram analysis of inflammation. (A3, B3, C3): Representative WLB,AFB imaging and RGB histogram analysis of LGD inflammation. (A4, B4, C4): Representative WLB,AFB imaging and RGB histogram analysis of HGD. (A5, B5, C5): Representative WLB,AFB imaging and RGB histogram analysis of invasive carcinoma. HGD, high‐grade preinvasive; LGD, low‐grade preinvasive.

### The diagnostic evaluation of WLB and/or AFB

In the study, 114 cases were diagnosed as positive by WLB, which included 102 true‐positive cases and 12 false‐positive cases; 104 cases were diagnosed as negative by WLB, which included 62 false‐negative cases and 42 true‐negative cases. The sensitivity (Se), specificity (Sp), positive predictive value, and negative predictive value were 62.2%, 77.8%, 89.5%, and 40.4%, respectively.

In total, 173 cases were diagnosed as positive by WLB associated with AFB, which included 151 true‐positive cases and 22 false‐positive cases, while 45 cases were diagnosed as negative by WLB + AFB, which included 13 false‐negative cases and 32 true‐negative cases. The Se, Sp, positive predictive value and negative predictive value were 92.1%, 59.3%, 87.3%, and 71.1%, respectively.

Comparing the sensitivities of the two methods using chi‐square test, we found a significant difference (*P* < 0.01) between WLB associated with AFB (92.1%) and WLB alone (62.2%). There was also a significant difference (*P* < 0.05) in the specificity of finding positive lesions between WLB associated with AFB(59.3%)and WLB alone(77.8%)(Table 2).

**Table 2:** The diagnostic evaluation of WLB and AFB associated with WLB

	WLB+AFB	WLB
Sensitivity	92.1% (151/164)**	62.2% (102/164)
Specificity	59.3% (32/54)*	77.8% (42/54)
Positive predictive value	87.3% (151/173)	89.5% (102/114)
Negative predictive value	71.1% (32/45)**	40.4% (42/104)

AFB, autofluorescence bronchoscopy; WLB, white light bronchoscope. The AFB associated with WLB group compared with the WLB group, *P <* *0.05, **P <* *0.01.

### Relations between pathological diagnosis and AFB image quantitative values (RGB system)

Test results of R/G, R/B, and G/B values in all pathological groups are shown in Table 3. Mean and standard deviation (SD) of H, S, and V values are shown in pathological groups (Table 4).

**Table 3:** R/G___R/B___G/B values in the different groups

Variables	Groups	*N*	Mean ± SD
R/G	Invasive carcinoma	150	1.81 ± 0.35
	HGD	14	1.58 ± 0.30
	LGD	9	1.27 ± 0.15
	Inflammation	32	1.34 ± 0.32
	Normal	13	1.09 ± 0.22
R/B	Invasive carcinoma	150	1.47 ± 0.15
	HGD	14	1.47 ± 0.11
	LGD	9	1.41 ± 0.15
	Inflammation	32	1.44 ± 0.11
	Normal	13	1.49 ± 0.11
G/B	Invasive carcinoma	150	0.84 ± 0.19
	HGD	14	0.96 ± 0.17
	LGD	9	1.13 ± 0.21
	Inflammation	32	1.14 ± 0.33
	Normal	13	1.44 ± 0.39

HGD, high‐grade preinvasive; LGD, low‐grade preinvasive.

**Table 4:** HSV values mean and SD

Variables	Groups	*N*	Mean (M)	Standard deviation (SD)
H	Invasive carcinoma	150	0.78	0.36
	High‐grade preinvasive (HGD)	14	0.64	0.45
	Low‐grade preinvasive (LGD)	9	0.37	0.45
	Inflammation	32	0.42	0.42
	Normal	13	0.13	0.07
S	Invasive carcinoma	150	0.44	0.09
	High‐grade preinvasive (HGD)	14	0.37	0.08
	Low‐grade preinvasive (LGD)	9	0.30	0.07
	Inflammation	32	0.36	0.07
	Normal	13	0.35	0.09
V	Invasive carcinoma	150	0.60	0.20
	High‐grade preinvasive (HGD)	14	0.59	0.20
	Low‐grade preinvasive (LGD)	9	0.63	0.20
	Inflammation	32	0.66	0.23
	Normal	13	0.57	0.21

### Correlation between R/G value and pathological diagnosis

There were significant differences between the R/G values in the invasive carcinoma group and in the HGD group as well as the LGD, normal bronchial mucosa and inflammation groups.

In addition, there were statistical differences between the HGD group and the LGD group as well as normal bronchial mucosa and inflammation groups.

The results showed that R/G values were different among groups and can be used to discriminate between benign and malignant lesions and identify HGD with benign diseases, as shown in Figure 2A.

**Figure 2:** Red, green, blue (RGB) ratio and HSV of AFB in the different groups *compared with invasive carcinoma, *P* < 0.05; **compared with invasive carcinoma, *P* < 0.01, △compared with HGD,* P* < 0.05; △△compared with HGD,* P* < 0.01; ^++^compared with LGD,* P* < 0.01; ^#^compared with inflammation, *P* < 0.05; ^##^compared with inflammation, *P* < 0.01; HGD, ^#^high‐grade preinvasive; LGD, ^#^low‐grade preinvasive. AFB, autofluorescence bronchoscopy.

### Correlation between R/B value and pathological diagnosis

There were no significant differences in R/B value between groups of invasive carcinoma, HGD, LGD, inflammation, and normal bronchial mucosa, as shown in Figure 2B.

### Correlation between G/B value and pathological diagnosis

There were significant differences in G/B value between the normal bronchial mucosa group and the other groups (*P* < 0.001) (Fig. 2C). The *P* values of G/B value between normal bronchial mucosa group and inflammatory group, between normal bronchial mucosa group and HGD group, and between normal bronchial mucosa group and invasive carcinoma group were all <0.001, which is of statistical significance.

Furthermore, there were significant differences between invasive carcinoma and normal bronchial mucosa group, inflammation group, and LGD group (*P* < 0.001).

The results indicated that G/B value was an ideal index for measurement of normal bronchial mucosa, and can also be used for discriminating between invasive carcinoma and benign lesions.

### Correlation between HSV value and pathological diagnosis

H values of fluorescence images in these groups are shown in Figure 2D. H values were significantly different in invasive cancer compared to LGD group (*P* = 0.002), inflammation group (*P* = 0.000), and normal bronchial mucosa group (*P* = 0.000). H values between HGD and normal groups were significantly different (*P* = 0.000). H values between inflammation and normal groups were different (*P* = 0.016). Results showed that H values could better differentiate invasive cancer and benign disorders. There was statistical difference between other groups. S values of fluorescence images in these groups are shown in Figure 2E. S values between invasive cancer and HLD (*P* = 0.004), LGD (*P* = 0.000), inflammation (*P* = 0.000), and normal groups (*P* = 0.000) were significantly different. S values between HGD and LGD groups were statistically different (*P* = 0.033). V values of fluorescence images in these groups are shown in Figure 2F. There was no statistical difference in V values between groups and there was no obvious value in clinical application.

### ROC analysis and the cutoff value

R/G value can be used to distinguish benign from malignant diseases, and the ROC curve related to detection of pathological diagnosis for benign and malignant diseases was made based on data obtained in the study, with the area under the curve being 0.857. If R/G value of 1.485 was taken as cutoff value, the diagnostic sensitivity would reach 82.3% and the specificity would reach 80.5%, as shown in Figure 3.

**Figure 3:** ROC curve of R/G value for detection of benign and malignant lesions.

Therefore, the value can act as an evaluation index to be applied in clinical practice of AFB for discrimination between benign and malignant lesions.

## Discussion

AFB has provided certain help for the diagnosis of central‐type lung cancer compared with conventional WLB and precancerous lesions 11, 12, 13, 14. Currently, most of overseas studies have reported that the sensitivity of AFB alone or in combination with WLB was higher in detecting precancerous lesions and cancerous tissues than that of WLB alone 15, 16, 17, 18, 19, 20, 21. However, many factors, such as the friction damage of airway wall caused by bronchoscopy in the process, airway mucosal inflammation, oral anticoagulation, taking photosensitizing drugs within 3 months, and cytotoxic chemotherapy undergone within 6 months may lead to false‐positive results in AFB 11.

Although AFB associated with WLB seems to significantly improve the sensitivity to detect intraepithelial neoplasia, the specificity is still lower than WLB alone 16.Therefore, a more effective method was introduced in this study which was able to improve the specificity of AFB by further analysis of AFB image and quantification of relevant indicators. The correlation between different quantitative indicators and diseases was made to obtain more accurate diagnosis and identify the diseases.

RGB Space Hue Analysis is an international standard about hue defined by International Electrotechnical Commission (IEC) that obtains various colors through changes of the three color channels of red, green, and blue (RGB) and their mutual superposition. This system is currently widely used in image processing and digital media. Yoko Kusunoki et al. firstly used the ratio of RGB hue space to identify benign and malignant diseases in 2000, and the research discovered that red/green = 0.53 was the boundary for the identification of benign and malignant diseases using LIFE system 22. The study also found that, there were differences in R/G value between the invasive carcinoma group and the HGD, LGD, normal bronchial mucosa, and inflammation groups. There were also R/G value differences between the HGD group and the LGD, normal bronchial mucosa and inflammation groups, and significant differences between the HGD group and the normal bronchial mucosa group. Kyoko Nakanishi et al. 23 made AFB image analysis for 288 biopsy specimens using PDS‐2000 system and found that the ratio of R/G was significantly higher in severe dysplasia and cancer, which was of statistical significance compared to benign lesions such as inflammation. Pyng Lee et al. 8 studied AFB using Onco‐LIFE system through multi‐center collaboration and found R/G could significantly distinguish benign diseases from malignant diseases. If the R/G value was chosen as 0.54, the sensitivity would reach 85% and the specificity would reach 80%.

Although some scholars have obtained results of large randomized controlled trials for AFB images of RGB system, the conclusion still lacks commonality due to different equipment vendors, light source, light wavelength range, and chromatography continuity. As for the AFB system OLYMPUS, especially for populations in China, there is no clear research that has obtained similar conclusions of determining benign and malignant diseases with R/G value at present, while our study has made a preliminary exploration in this area.

Furthermore,the present explorative study analyzed and investigated the application of autofluorescence bronchoscopy image in HSV System, and quantified image information to facilitate clinical practice. HSV is a representation of color space and represents colors using three basic properties of color: hue, saturation, and value. HSV is a color model toward visual perception. Since HSV can reflect the human perception and identification to color better, it is very suitable for image processing 10. This quantified indicator more objectively and accurately guides clinical bronchoscopy. Judgment of the nature of target lesions by objective and quantified HSV values facilitates the diagnosis of diseases of patients and the operations of clinical bronchoscopy, and subjective factors could be avoided. Results showed that H values in autofluorescence images could better differentiate benign and malignant diseases. As an indicator for judging benign and malignant diseases, H value will effectively improve the positive rate of AFB, guide clinical operations, and avoid the influence of other factors.

However, we differentiated benign diseases (such as inflammation) with malignant diseases through quantitative analysis of autofluorescence bronchoscopy (AFB) images in different types of diseases in our study. With the promotion of quantitative method of AFB and development of scientific technologies, the fluorescence intensity at different pathological stages in the development of lung cancer will be quantified, enabling AFB to play a greater role in the early diagnosis of lung cancer, specification of the disease extent, and assessment of local cancer degree.

In addition, with in‐depth study of excitation light source and image processing of AFB and further improvement of the imaging system, AFB will play a more important role and be of greater clinical significance in terms of detection and diagnosis of bronchopulmonary cancer.

## Conflict of Interest

The authors declare no conflicts of interest.
